# Chemical Fingerprint Profiles and Pharmacodynamic Investigation for Quality Evaluation of Moxa Smoke by UHPLC in a Rat Model of Superficial Infection

**DOI:** 10.1155/2021/9929596

**Published:** 2021-07-31

**Authors:** Yanling Wang, Shengbing Wu, Leijing Chen, Guo Xu, Xiaoxiao Wang, Jie Wu, Bin Wang, Meiqi Zhou

**Affiliations:** ^1^Key Laboratory of Xin'an Medicine of the Ministry of Education, Anhui University of Chinese Medicine, Hefei, China; ^2^Key Laboratory of Acupuncture and Moxibustion Foundation and Technology of Anhui Province, Anhui University of Chinese Medicine, Hefei, China; ^3^Bozhou Institute of Traditional Chinese Medicine, Anhui Academy of Chinese Medicine, Bozhou, China

## Abstract

**Introduction:**

Moxibustion, a traditional Chinese medicine technique, involves the use of moxa smoke from *Folium Artemisia argyi* to treat various disorders, especially superficial infections. However, there is a higher health risk for people exposed to high levels of moxa smoke for extended durations. Here, we report the first ultra-high-performance liquid chromatography (UHPLC) fingerprint profiles and pharmacodynamic evaluation of moxa smoke, as well as evaluation of its aqueous solution on a rat model of superficial infection.

**Methods:**

A novel method for moxa smoke fingerprint profiling was developed using UHPLC under characteristic wavelength. Chromatographic peaks were further analyzed by ultra-high-performance liquid chromatography quadrupole-time-of-flight mass spectrometry (UHPLC-QTOF/MS). 12 sample batches obtained from various Chinese provinces were then analyzed using similarity evaluation, clustering analysis, and principal component analysis. The pharmacodynamics of moxa smoke and moxa aqueous solution were investigated on a rat model of acute skin wound infection.

**Results:**

UHPLC fingerprint profiles of 12 batches of moxa smoke were generated at 270 nm wavelength and 21 chromatographic peaks extracted as common peaks. Similarity between the 12 batches ranged from 0.341 to 0.982. Based on cluster analysis, the 12 batches of moxa smoke samples were clustered into five groups. Principal component analysis showed that the cumulative contribution of the three principal components reached 90.17%. Eigenvalues of the first, second, and third principal components were 10.794, 6.504, and 1.638, respectively. The corresponding variance contribution rates were 51.40%, 30.97%, and 7.80%, respectively. Pharmacological analysis found that wound healing was slow in the model group relative to the mupirocin ointment, moxa smoke, and aqueous moxa smoke solution groups. Histological analysis revealed markedly reduced tissue inflammation in rats treated with moxa smoke or its aqueous solution.

**Conclusions:**

Moxa smoke and its aqueous solution significantly promote wound healing upon superficial infection. A novel quality control method for moxa smoke was established and evaluated for the first time. As its main effects are unchanged, the transformation of moxa smoke into aqueous moxa smoke improves safety and is a simple and controllable process.

## 1. Introduction

Traditional Chinese medicine (TCM) has been widely used in many Asian countries, especially in China, to treat various diseases for millennia [1, 2]. Moxibustion, usually using mugwort from *Folium Artemisia argyi* has antibacterial and antiseptic effects and is used in TCM for the treatment and prevention of illness through activation of self-healing [3]. Moxibustion with fumigation, also called fumigated moxibustion, is recorded in 52 disease formulae. It has a long history in China with good therapeutic effects against surgical infections [4, 5]. However, during fumigation moxibustion, extended exposure to high levels of moxa smoke from mugwort sticks poses a higher health risk [6–10]. Thus, it is necessary to develop effective moxa smoke quality control procedures to ensure its efficacy and safety.

Moxa smoke therapeutic benefits are attributed to numerous active components, which have not been fully elucidated [11, 12]. Additionally, analysis and identification of moxa smoke active components is challenging due to the diversity and complexity of TCM compounds. TCM fingerprinting is a simple and effective method of evaluating TCM quality and allows a comprehensive detection of a sample's main components [13, 14]. Coupling UHPLC fingerprints with the Mass Spectrometer (MS) technique allows the evaluation of the complex composition of TCM.

We previously developed a Gas Chromatography coupled with Mass Spectrometer (GC-MS) method for qualitative identification of volatile oils and burnt smoke in *Artemisia argyi*, which allowed preliminary quality evaluation of moxa smoke [15]. In 2016, we invented a new equipment of collecting moxa smoke, which has been patented by the national intellectual property administration of the People's Republic of China (patent no. ZL 201610105632.3). We recently found that *Artemisia argyi* volatile oils have good antibacterial effects and more recently, progress in *Artemisia argyi* genomics has been made [16, 17]. Here, we report a fingerprint method based on UHPLC and MS for comprehensively evaluating moxa smoke quality [18–21]. Converting moxa smoke into an aqueous form will lower the risk posed by exposing patients to moxa smoke. Moxa smoke fingerprint profiles were constructed, and the common peak identified by UHPLC and MS was selected. Finally, the therapeutic effect of moxa smoke and aqueous moxa smoke on superficial infections was evaluated using animal experiments.

## 2. Experiments

### 2.1. Materials and Reagents

The 12 batches of mugwort stick (S_1_–S_12_) were purchased from Nanyang Yilejia Mugwort Products Co., LTD. (batch no: 20200102), Nanyang Zhanfang Artemisia argyi Co., LTD. (batch no: 20190102), Nanyang Hanyi Trading Co., LTD. (batch no: 20200415), Nanyang Hanai Mugwort Products Co., LTD. (batch no: 20191205), Pingli Zhonghuang Wild Mugwort Scientific Research Industry and Trade Co., LTD. (batch no: 20191205), Qingdao Zhenaitang Traditional Chinese Medicine Technology Co., LTD. (batch no: 20180311), Qichun Haofan Qi Ai Products Co., LTD. (batch no: 20200403), Jiangsu Kangmei Pharmaceutical Co., LTD. (batch no: 20190916), Anhui Lvyingtang Cailong Mugwort Pharmaceutical Co., LTD. (batch no: 1200202), Linxiang Huxiang Ai Biotechnology Co., LTD. (batch no: 20181201), Yantai Aixin Medical Equipment Co., LTD. (batch no: 20200301), and Ningxia Ze Aitang Biotechnology Co., LTD. (batch no: 20200504), respectively. Chromatographic methanol and acetonitrile were purchased from MERCK. Deionized water was prepared using a Milli-Q purification system (Millipore). Ulai was purchased from Shanghai yuanye Bio-Technology Co., Ltd. Ammonium acetate and sodium sulfide, including nine hydrate, were analytically pure. The isoflurane was obtained from RWD Life Science Co., Ltd. Mupirocin ointment was purchased from Hubei Renfu Chengtian Pharmaceutical Co., LTD. (batch no: 20200202).

### 2.2. Animals and Experimental Design

#### 2.2.1. Animals

Ethical approval for animal use was granted by the Committee on the Ethics of Animal Experiments of Anhui University of Chinese medicine. Specific Pathogen Free (SPF) grade, male Sprague Dawley (SD) rats (200–250 g) were purchased from the breeding center of Anhui Medical University (License No. SCXK (Lu) 20190003). Animals were housed individually at 18–22°C, 40–60% humidity, and 12 h light/dark cycle with *ad libitum* access to food and water and minimal environmental noise. All efforts were made to minimize animal suffering in accordance with the principles of the Animal Care and Use Committee, Anhui University of Chinese Medicine.

#### 2.2.2. Bacterial Strain

*Staphylococcus aureus* was obtained from the Laboratory of Microbiology and Biochemistry, College of Integrated Traditional Chinese and Western Medicine, Shaoquanhu Campus, Anhui University of Chinese Medicine.

#### 2.2.3. Animal Groups

All rats were randomly split into five groups, namely, the normal group, model group, mupirocin ointment group, moxa smoke group, and aqueous moxa smoke group (*n* = 7). A model of skin wound infection was established in all rats except the normal group according to the work in [22]. Briefly, rats were weighed and placed in induction boxes and anesthetized. They were then transferred to an induction box and placed on fixation plates for operation. Next, a large area of primary hair was removed from the back using a hair pusher, followed by complete hair removal with 10% sodium sulfide nine hydrate. The hair-removed section was then rinsed with normal saline and dried. After hair loss, rats were placed on a treatment table with the back facing up and the back skin disinfected with iodine volts. A 1.5 cm (diameter) incision was then made in the middle of the spine, and tweezers were used to injure the skin at the incision until the muscle layer was destroyed. The wound was then swabbed with a cotton swab and 80 *μ*L (2.53 × 10^9^) of *Staphylococcus aureus* solution was introduced into the wound. A sterile application was then used to close the wound, ensuring contact between the bacteria solution and skin wound. After waking from anesthesia, rats were placed in a feeding cage with independent ventilation. After 48 h, a significant pyogenic formation was observed on the backs, indicating successful establishment of a rat model of skin wound infection. Model group rats received an equal amount of solvent.

#### 2.2.4. Administration Method

The normal and model group received saline debridement, respectively. The mupirocin ointment group was daubed with 0.30 mL/100 g of mupirocin ointment. The moxa smoke group was daubed with 0.30 mg/100 g, 0.45 mg/100 g, and 0.6 mg/100 g of moxa smoke solution. The administration method was carried out once daily for 7 days in a row. Changes in diet, body weight, and wound size were observed during the modeling period.

#### 2.2.5. Pharmacodynamic Evaluation

On the 16^th^ day, all rats were deeply anesthetized with isoflurane (3 mL/kg). Body weight, diet, and wound healing were monitored during the 7-day treatment. Wound tissues were obtained and fixed in 10% neutral formalin, and histological analysis conducted using Hematoxylin-Eosin (H&E) staining.

### 2.3. Analysis and Identification for Moxa Smoke

#### 2.3.1. Moxa Smoke Solutions

One mugwort stick (about 20 g) from the Henan region, China, was burnt to generate moxa smoke. An atomizer with 20 mL deionized water was used to atomize incessantly at a speed of 3 mL/min to provide fogdrop (particle diameter = 3.9 *µ*m). Moxa smoke and fogdrop were mixed in a 3 L container. The whole process takes about 40 min. Aqueous moxa smoke solution S_1_ was then prepared in a 25 mL volumetric flask. Aqueous moxa smoke solutions for the other 11 sample solutions (S_2_–S_12_) were prepared in the same way. The solution was then filtered on a 0.22 *μ*m microporous membrane, and the solutions were stored at 4°C until analysis. 50 and 75% aqueous moxa smoke solutions were then prepared by diluting solutions S_2_–S_12_ with distilled water.

#### 2.3.2. Selection of Ultraviolet (UV) Absorption Wavelength of Moxa Smoke Solutions

Objectively setting the UV detection wavelength is very important in UHPLC fingerprints analysis. So, we analyzed all 12 sample batches at full wavelength by scanning with a UV spectrophotometer and recording their absorbance data.

#### 2.3.3. UHPLC-UV Method

All analyses were conducted on an Agilent Eclipse Plus C_8_ (2.1 × 100 mm, 1.8 *µ*m) chromatographic column at column and sample chamber temperatures of 30°C and 10°C, respectively. UV wavelength was set at 270 nm. UHPLC mobile phase was comprised of A (water containing 0.1% ammonium acetate solution) and B (acetonitrile). The gradient was set as follows: 0–8 min, 99% A; 8–9 min, 99%–97% A; 9–12 min, 97% A; 12–13 min, 97%–95% A; 13–20 min, 95% A; 20–21 min, 95%–90% A; 21–26 min, 90% A; 26–32 min, 90%–60% A; 32–33 min, 60%–30% A; 33–35 min, 30% A; 35–36 min, 30%–99% A; and 36–40 min, 99% A. Optimal chromatographic results were obtained at a flow rate of 0.2 mL/min and a sample injection volume of 1.0 *μ*L.

#### 2.3.4. UHPLC-QTOF/MS Method

For UHPLC-QTOF/MS analysis, an ACQUITY I-Class UHPLC equipment coupled with a Xevo G2-XS QTOF/MS detector (Waters Corp.) via an electrospray interface was used. Mass spectrometry was performed in positive and negative ionization modes, and corresponding data were obtained between 200 and 600 m/z at a data acquisition rate of 0.5 s. For accuracy, m/z values of all ions acquired in the QTOF/MS were real-time adjusted by Lock Spray, with leucine-enkephalin used as the lock mass compound for the positive ionization mode ([M + H]^+^: m/z 556.2771) and negative ionization mode ([M − H]^−^: m/z 554.2615). Components of all analyzed samples generally produced molecular adduct ions such as [M + H]^+^ or [M−H]^−^, which were further fragmented by collision energy application.

## 3. Results and Discussion

### 3.1. Collection Method of Moxa Smoke

12 batches of mugwort stick from 9 different Chinese regions were burnt to generate moxa smoke. Next, moxa smoke aqueous solution was obtained by mixing the moxa smoke with fogdrop from an atomizer (Figure 1). The use of aqueous moxa smoke may avoid the risk posed to the patient by exposure to moxa smoke.

### 3.2. Pharmacodynamic Evaluation

#### 3.2.1. Monitoring Wound Healing

The flowchart is shown in Figure 2(a). The rat model of skin wound infection was established in 7 days. In the 9^th^ to 12^th^ days, animals in the normal group gained weight steadily. Animals in the model group significantly lost weight in this period and had loose stools. Their wounds did not heal naturally. In contrast, rats in the treated groups, including mupirocin ointment, moxa smoke, and aqueous moxa solution groups, slightly lost weight and had loose stools. On the 13^th^ day, the rats' diet in the treated group gradually improved and weight rose gradually. On the 16^th^ day, the wound areas had significantly reduced before and after treatment (Figures 2(b)–2(c)), showing the moxa smoke could promote the wound healing. Relative to the moxa smoke group, the aqueous moxa smoke group exhibited similar effects.

#### 3.2.2. Pathological Tissue Section Changes

After 7 days of treatment, H&E pathological analysis (Figure 2(d)) did not uncover inflammatory cell infiltration and revealed that skin epithelial cells were arranged neatly. The wound in the model group was moist, with more exudate and less obvious contraction. Pathological analysis showed no granulation tissue growth. However, a large number of leukocytes, eosinophils, neutrophils, and other inflammatory cells infiltrated the superficial, deep, and subcutaneous skin tissues.

### 3.3. Establishment of UHPLC Fingerprint of Moxa Smoke

Here, chemical fingerprinting was used, and it is an important technique for the quality evaluation of natural products [23]. Additionally, the identification of the chemical fingerprint of TCMs involves a variety of extraction methods, for example, sonication, reflux, presoaking, pretreatment, and hydrolysis [24]. The fingerprint profiles of 12 batches of moxa smoke (extracted using the pretreatment) were established through using chemometric methods. Specifically, because full wavelength scanning revealed the maximum absorption wavelength for moxa smoke solution as 270 nm (Figure 3), we set UHPLC detection wavelength at 270 nm. Samples S_1_–S_12_ were analyzed using the optimal conditions outlined in Section 2.3.3, and data were analyzed using similarity evaluation software of Chinese medicine chromatogram fingerprint (2012 Version) using the sample **S**_**1**_ reference map. The median method was used, and time window was set at 0.1 min. Next, chromatogram peaks were analyzed by automatic matching after multipoint correction, and finally, the moxa smoke UHPLC fingerprint was established (Figure 4).

#### 3.3.1. Investigation of the Fingerprint Methodology

(1) Precision test: 1.0 *μ*L sample **S**_**1**_ was injected 6 times, and resulting chromatograms were recorded. Relative retention time and relative peak area of each common peak were then investigated. Taking peak **12** as the reference peak, this analysis showed the RSD of the relative retention time and relative peak area were <1.7 and <3.8%, respectively, indicating good UHPLC precision.

(2) Stability test: 1.0 *μ*L of sample **S**_**1**_ was injected at 0, 2, 6, 4, 8, 10, 12, and 24 h, and chromatograms were recorded. Relative retention time and relative peak area for each common peak were then investigated. Taking peak **12** as the reference peak, this analysis showed that the RSD of the relative retention time and the relative peak area was <2.0 and <1.35%, respectively, indicating good stability for sample **S**_**1**_ at 24 h.

(3) Repeatability test: 1.0 *μ*L of sample **S**_**1**_ was injected 6 times, and chromatograms were recorded. Relative retention time and relative peak area for each common peak were then investigated. Taking peak **12** was taken as the reference peak, and the results showed the RSD of the relative retention time and the relative peak area was <0.6 and <3.6%, respectively, indicating the method's repeatability was fine.

#### 3.3.2. Selection and Identification of Common Peaks

Because the UHPLC chromatogram of the 12 batches of moxa smoke solutions showed that the area of peak **12** was moderate and its retention was stable, it was selected as the reference peak. Next, the common pattern diagram of moxa smoke fingerprint chromatograms at 270 nm was exported from the similarity evaluation software (Figure 5). Data of the common peaks of 12 batches of moxa smoke decoction at 270 nm were also exported from the software. The results showed 33 chromatographic peaks were found in fingerprint chromatograms and 21 peaks could be matched as common peaks with relative retention times <1.21%.

QTOF/MS spectra were detected in both positive and negative ion modes. Components in the moxa smoke sample generally produced molecular adduct ions, such as [M + H]^+^ or [M − H]^−^, which were then fragmented using collision energy. Based on the past study sand fragmentation behavior, common peaks were identified by QTOF/MS spectra. Peaks **2**, **5**, **7**, **8**, **9**, **10**, **12**, **14**, **18**, and **19** were ascribed to azulene **(2)**, furfuryl alcohol **(5)**, cineole **(7)**, 3,5-dimethyl-2-cyclohexen-1-one **(8)**, *α*-thujone **(9)**, o-cresol **(10)**, catechol **(12)**, eugenol **(14)**, 4-ethylphenol **(18)**, and 1,2-benzenediol,5-(1,1-dimethylethy)-3-methyl-**(19)** (Figure 6) (Table 1).

As well known, phenols generally exhibit antioxidant activity. In this study, we found that there are some phenolic compounds in the combustion of *Artemisia argyi*, for instance, o-cresol (peak **10**), catechol (peak **12**), eugenol (peak **14**), and 4-ethylphenol (peak **18**). So, they may be closely related to the substance basis of the efficacy of moxibustion in the treatment of superficial infectious diseases.

#### 3.3.3. Evaluation of Similarity

Similarity results of 12 moxa smoke solution batches at 270 nm were obtained from the Similarity Evaluation System of Traditional Chinese medicine chromatographic fingerprint (2012 version) and ranged from 0.341 to 982 (Table 2). Except for the **S**_**2**_, **S**_**3**_, **S**_**4**_, and **S**_**12**_ samples, sample similarities were >0.9.

#### 3.3.4. Clustering Analysis

With the peak areas of 21 common peaks as the standard, Statistical Product and Service Solutions (SPSS) 23.0 software was used, and the method of intergroup mean association was adopted. The included angle cosine was selected by the distance formula of sample similarity to systematically cluster the 12 batches of moxa smoke samples (Figure 7).

Based on cluster analysis, the 12 moxa smoke sample batches were clustered into 5 groups with **S**_**3**_, **S**_**4**_, **S**_**5**_, **S**_**6**_, and **S**_**9**_ clustered into class I, **S**_**2**_, **S**_**7**_, **S**_**8**_, and **S**_**12**_ clustered into class II, **S**_**10**_ clustered into class III, **S**_**11**_ clustered into class IV, and **S**_**1**_ clustered into class V.

#### 3.3.5. Principal Component Analysis (PCA)

SPSS 23.0 was used to standardize the original data, and the characteristic root, and the contribution rate of principal components was used as the basis for selecting principal components for principal component analysis. The top 3 principal components whose eigenvalues were >1 were selected for principal component analysis on 21 common peaks (variables) of 12 samples (observed objects). This analysis showed that the cumulative contribution of the 3 principal components reached 90.17%. The eigenvalues of the 1^st^, 2^nd^, and 3^rd^ principal components were 10.794, 6.504, and 1.638, respectively. The corresponding variance contribution rates were 51.40%, 30.97%, and 7.80%, respectively. The coordinate system was established with the 1^st^, 2^nd^, and 3^rd^ principal components, respectively, and PCA 3D maps for all samples were obtained after projection (Figure 8). Thus, the 21 common peaks can be divided into 3 categories.

After analysis, we obtained the results of the common factor load matrix after rotation (Table 3), indicating that each load amount represents the correlation coefficient between the principal component and corresponding variable. The component model was then obtained on SPSS 23.0 as follows:

  A_1_ = 0.007F_1_ + 0.065F_2_ − 0.017F_3_ + 0.070F_4_ - 0.032F_5_ + 0.089F_6_ + 0.072F_7_ + 0.079F_8_ + 0.059F_9_ + 0.018F_10_ + 0.091F_11_ + 0.074F_12_ − 0.015F_13_ + 0.090F_14_ + 0.040F_15_ − 0.037F_16_ + 0.065F_17_ + 0.086F_18_ + 0.088F_19_ + 0.088F_20_ − 0.085F_21_
  A_2_ = 0.139F_1_ + 0.040F_2_ − 0.143F_3_ + 0.038F_4_ + 0.140F_5_ − 0.020F_6_ − 0.042F_7_ − 0.049F_8_ + 0.116F_9_ + 0.148F_10_ − 0.002F_11_ + 0.033F_12_ + 0.138F_13_ − 0.020F_14_ + 0.122F_15_ + 0.121F_16_ + 0.026F_17_ + 0.003F_18_ + 0.004F_19_ + 0.005F_20_ + 0.020F_21_
  A_3_ = 0.021F_1_ + 0.047F_2_ + 0.082F_3_ + 0.289F_4_ + 0.076F_5_ + 0.114F_6_ + 0.323F_7_ + 0.225F_8_ + 0.077F_9_ + 0.013F_10_ − 0.022F_11_ − 0.302F_12_ − 0.095F_13_ − 0.107F_14_ − 0.035F_15_ + 0.120F_16_ − 0.401F_17_ − 0.073F_18_ − 0.184F_19_ + 0.089F_20_ − 0.042F_21_

Components 1–3 represent 3 principal components, respectively. F_1_–F_21_ represent normalized relative peak area data for each chromatographic peak. Of the 3 principal components, component 1 is the peak with the largest eigenvalue. The top 5 variable coefficients in the 1^st^ principal component were 0.091, 0.090, 0.089, 0.088, and 0.086.

Peaks **2**, **4**, **6–9**, **11–12**, **14**, and **17–20** had obvious positive -phase load in the first principal component, indicating that the characteristic value of the 1^st^ principal component increases with the increase of its specific gravity (Table 2). Similarly, peaks **1**, **3**, **5**, **9–10**, **13**, and **15–16** are the main determinants in the 2^nd^ principal component. In the 3^rd^ principal component, peaks **3–9**, **16**, and **20** have obvious positive-phase loads.

#### 3.3.6. Orthogonal Partial Least Squares Discriminant Analysis (OPLS-DA)

In order to further illustrate the weight of the potential chemical index components in moxa smoke solutions, we utilized OPLS-DA to analyze the variables of the peak area, as shown in Figure 9. The result showed that 12 batches of samples were divided into five categories, which were consistent with the results of clustering analysis. In addition, 21 components were further screened based on the variable importance of the projection (VIP) value for selecting the markers (Figure 10). VIP represents the difference of variables. When the VIP value is greater than 1.0, it means that the component plays a vital role in the differentiation. Based on the OPLS-DA, the VIP values of peaks 11, 14, 6, 20, 19, 18, 21, 8, 12, 7, and 4 were >1.0. The three components, namely, eugenol (peak **14**), 4-ethylphenol (peak **18**), and 1, 2-benzenediol,5-(1,1-dimethylethyl)-3-methyl (peak **19**), had a great influence on the differentiation.

## 4. Conclusions

Here, novel UHPLC fingerprints of moxa smoke solutions at a characteristic 270 nm wavelength were developed for the first time. 21 common peaks in the fingerprint chromatograms were obtained through the similarity evaluation system. Combined with UHPLC-QTOF/MS in both the positive and negative ion mode, 10 common peaks in the 21 common peaks were identified or tentatively characterized based on their *t*_R_, UV spectra, MS spectra, and previous reports. Similarity, clustering analysis, and principal component analysis showed that mugwort sticks purchased from Henan, Shangdong, Shangxi and Jiangsu, Hunan, Anhui, and Ningxia regions of China have major differentiation. Additionally, pharmacodynamic analysis indicated both moxa smoke and its aqueous solution may significantly promote healing of wounds with superficial infection. Our data indicate that because its main effects are unchanged, transformation of moxa smoke into aqueous moxa smoke not only reduces harm but also is a simple and controllable procedure. Importantly, our findings offer reference for clinical applications.

## Figures and Tables

**Figure 1:** Collected equipment of the moxa smoke.

**Figure 2:** The evaluation of pharmacodynamics experiments.

**Figure 3:** The UV absorption spectrum of 12 batches of moxa smoke solutions.

**Figure 4:** The UHPLC fingerprints of moxa smoke solutions at 270 nm.

**Figure 5:** The common pattern diagram of moxa smoke fingerprints at 270 nm.

**Figure 6:** The structures of 10 common peaks identified by QTOF/MS.

**Figure 7:** Cluster analysis diagram of 12 batches of moxa smoke.

**Figure 8:** Picture of principal component score.

**Figure 9:** OPLS-DA score of 12 batches of moxa smoke samples.

**Figure 10:** The VIP value for classification of common peaks from12 batches of moxa smoke samples.

**Table 1:** Identification of chemical constituents of moxa smoke by UHPLC-QTOF/MS.

No.	*t*_R_/min	Formula	Parent ion	Theoretical mass (m/z)	Measured mass (m/z)	Identification	Ref
1	1.55	C_10_H_8_	[M−H]^−^	128.06	128.00	Azunlene	[25]
2	4.36	C_5_H_4_O_2_	[M−H]^−^	98.09	98.92	Furfurl alcohol	[25]
3	5.36	C_7_H_8_O	[M−H]^+^	108.06	108.08	o-Cresol	[25]
4	6.84	C_6_H_6_O_2_	[M−H]^+^	110.11	110.09	Catechol	[25]
5	8.12	C_10_H_12_O_2_	[M−H]^+^	164.08	164.08	Eugenol	[26]
6	8.97	C_8_H_12_O	[M−H]^+^	124.09	124.09	3,5-Dimethyl-2-cyclohexen-1-one	[27]
7	11.84	C_11_H_16_O_2_	[M−H]^+^	180.11	180.09	1,2-Benzenediol,5-(1,1-dimethylethyl)-3-methyl	[27]
8	14.36	C_10_H_16_O	[M−H]^+^	152.12	152.10	-*α*-Thujone	[26]
9	24.94	C_8_H_10_O	[M−H]^−^	122.07	122.03	4-Ethylphenol	[25]
10	38.35	C_10_H_18_O	[M−H]^+^	154.14	154.98	Cineole	[28, 29]

**Table 2:** The similarity results of 12 batches of moxa smoke decoction at 270 nm.

No.	S_1_	S_2_	S_3_	S_4_	S_5_	S_6_	S_7_	S_8_	S_9_	S_10_	S_11_	S_12_
1	1											
2	0.794	1										
3	0.669	0.779	1									
4	0.549	0.427	0.341	1								
5	0.983	0.789	0.661	0.532	1							
6	0.912	0.629	0.565	0.426	0.904	1						
7	0.97	0.817	0.728	0.502	0.969	0.902	1					
8	0.966	0.671	0.538	0.539	0.964	0.946	0.943	1				
9	0.966	0.732	0.565	0.565	0.969	0.891	0.959	0.979	1			
10	0.94	0.725	0.617	0.497	0.956	0.956	0.958	0.97	0.964	1		
11	0.979	0.786	0.661	0.548	0.981	0.899	0.98	0.968	0.985	0.961	1	
12	0.733	0.824	0.958	0.397	0.738	0.645	0.804	0.609	0.636	0.69	0.723	1

**Table 3:** Factor load matrix results.

Peak	Compound		
	1	2	3
F1	0.007	0.139	0.021
F2	0.065	0.04	0.047
F3	−0.017	0.143	0.082
F4	0.07	0.038	0.289
F5	−0.032	0.14	0.076
F6	0.089	−0.02	0.114
F7	0.072	−0.042	0.323
F8	0.079	−0.049	0.225
F9	0.059	0.116	0.077
F10	0.018	0.148	0.013
F11	0.091	−0.002	−0.022
F12	0.074	0.033	−0.302
F13	−0.015	0.138	−0.095
F14	0.09	−0.02	−0.107
F15	0.04	0.122	−0.035
F16	−0.037	0.121	0.12
F17	0.065	0.026	−0.401
F18	0.086	0.003	−0.073
F19	0.088	0.004	−0.184
F20	0.088	0.005	0.089
F21	−0.085	0.021	−0.042

## Data Availability

The data used to support the findings of this study are available from the corresponding author upon request.
